# Evaluation of Pollution Status and Detection of the Reason for the Death of Fish in Chamo Lake, Ethiopia

**DOI:** 10.1155/2022/5859132

**Published:** 2022-04-27

**Authors:** Daniel Reddythota, Mosisa Teferi Timotewos

**Affiliations:** ^1^Faculty of Water Supply & Environmental Engineering, Arba Minch Water Technology Institute, Arba Minch University, Arba Minch, Ethiopia; ^2^Department of Water Engineering, Technical University of Berlin, Berlin, Germany

## Abstract

Chamo Lake is the third largest rift valley lake and one of the major economic sources for the communities in the Southern region, Ethiopia. The lake's quality is deteriorating due to the untreated wastewater, and sediment inflow resulting in the death of fish was observed during the dry season. The research aims to determine the water quality status using water quality indices, in addition to identifying the reason for the death of fish in the dry season in Chamo Lake. The water samples were drawn from 5 sampling points by composite sampling method during the dry and wet seasons of the year, and we analyzed 22 water quality parameters. Ammonia (14–23.6 mg/l), phosphates (0.30–1.10 mg/l), BOD (25.32–60 mg/l), COD (40–160 mg/l), and chlorophyll (19.64–31.87 *μ*g/L) concentrations were above the permissible limits, and DO (5.20–6.70 mg/l) was below the acceptable limit in the lake as per EPA standards concerning temperature. The values of both the water quality indices of CCMEWQI (13.90–18.40) and NSFWQI (38.59–49.63) indicated that the water quality was “poor” and “bad,” respectively. The death of fish might be due to high concentrations of ammonia and nutrients in the dry season.

## 1. Introduction

Surface water resources are most vulnerable to pollution due to their easy accessibility for the disposal of pollutants and wastewater. The surface water quality is pressured by point and nonpoint sources of pollution [1]. Anthropogenic activities such as industrialization [2], urbanization, agricultural runoff, construction activities, and domestic activities as well as natural activities such as climate change [3], soil erosion [4], and sedimentation will intensify water pollution [5] and water scarcity [6]. Water pollution causes diseases, water scarcity, mortality of aquatic life, and the environment that affects human life and hindrance to community development. The deteriorated water quality becomes toxic to the aquatic life and causes eutrophication, which affects the sustainability of lakes.

Over the past two decades, most of the water bodies in Ethiopia have become increasingly threatened due to pollution from different sources. Among freshwater resources, Lake Chamo is one of the major rift valley lakes in Ethiopia and is used for various purposes by semiurban and urban dwellers. Chamo Lake serves multiple purposes such as fisheries, agriculture, flood control, and tourism in the study area. Rapid urbanization and extensive anthropogenic activities enriched the pollution load in the lake. Conversely, rainfall events can furthermore accelerate the pollutant load due to sediment inflow, entry of stormwater, runoff from urban areas along with urban untreated domestic wastewater, as well as runoff from agricultural areas. Increased nutrient load causes Eutrophication of the lake [7, 8] leading to decrease fish production, loss of surrounding community economic sources (tourism and fish), and disappearance of the lake.

All the previous studies did not use water quality indices to find out the pollution status of the lake. During the dry season in 2018, fishes were dead and floating on the surface suddenly for a few days that was observed by the fishermen. No previous researchers investigated the reason for the death of fish. Inflows of various tributaries into the lakes have the possibility of lake contamination. In the assessment of surface water resources, water quality is important for the identification of pollutant circulation routes [9]. So it is essential to study the water quality, in addition to finding out the status of pollution by using water quality indices. Identification of pollution sources and developing an appropriate control approach [10] are essential to minimize pollution as well as enhance the sustainability of water resources. The sustainable management of water resources depends upon the monitoring and controlling of the processes of change [11].

This study aims to assess the pollution status of Chamo Lake by using two different water quality indices, in addition to identifying the reason for the death of fish in the lake. Besides, identify the possible pollution sources of the lake. This research work will be very useful for the researchers, those who are researching the river water quality, as well as the administrative authorities of water conservation.

## 2. Methodology

### 2.1. Description of the Study Area

The study area, Chamo Lake, is located at the coordinates of 5^0^50′59″ N; 37°33′54″ E in the Southern Nations, Nationalities, and People's Regional State (SNNPRS) of Ethiopia (Figure 1); Lake Anaya to the south, the Guge Mountains to the east, and nearby the town of Arba Minch with an altitute of 1,235 m above sea level. This lake is naturally separated from Lake Abaya by a 5 km-wide ridge with a vertical offset of approximately 60 m [12]. The catchment area of Lake Chamo is 1,109 km^2^, and the surface area is 329 km^2^. The rivers Kulfo, Sile, and Elgo are the main perennial rivers draining into the lake. Lake Abaya and Lake Chamo have been interconnected in the past, with water flowing from Lake Abaya into Lake Chamo via the Kulfo River, but the lakes were disconnected from 1980 until 2013 due to sediment deposition [13]. The climate in the catchment is defined as a humid to hot semitropical. The bimodal rainfall pattern of the catchment has two wet seasons (March to mid-June and mid-September to late November) and two dry seasons (December to mid-March and mid-June to mid-September). The mean annual rainfall and temperature were 1,351.8 mm and 23.9 C, respectively, in the study area. During the year, the average temperatures vary by 2.4°C. The evaporation is highest during March and July [14].

### 2.2. Hydrological Parameters

#### 2.2.1. Rainfall and Temperature

Rainfall and temperature will influence the water quality directly as well as indirectly. High rainfall causes to increase in the inflow of pollutants and sediment to affect the water quality of the water bodies. In contrast, high rainfall will reduce the toxicity of the pollutants due to dilution. High temperatures cause to increase in the evaporation rate so that the concentration of the pollutants will be increased. Rainfall and temperature data were collected over 15 years (2006–2020) from the National Meteorological Agency of Ethiopia and the National Remote Sensing Agency (NASA), USA (Figure 2).

### 2.3. Sample Site Selection and Sampling

The research team visited before sample collection to select the sampling points at Chamo Lake and selected five sampling points to survey in Chamo Lake for sample collection, namely, four samples from the peripheral and one sample from the centre part. The first sampling point was at Kulfo River entering point into Chamo Lake; the second sampling point was near the boat station; the third sampling point was a central point of the lake; the fourth sampling point was near Nechasar Park; and the fifth sample was collected at the farmland side. Sampling points were selected based on the inlets with their location, uses of the lake water and their location, and importance and magnitude of human influence in the peripheral and central areas of the lake.

Water samples were collected from the lake during the dry and wet seasons at five selected sampling sites with a 2 L sampler bottle. At each sampling site, we collected five subsamples around the sampling site at different spaces and mixed them in a bucket, and 2 L of the sample was filled in a sample bottle (space-interval composite sampling). The collected 2 L sample bottles were transported within a short period to the laboratory. Samples were analyzed in the Arba Minch Water Quality laboratory by standard methods [15] (Table 1).

### 2.4. Water Quality Analysis

The physicochemical and biological parameters, namely, temperature (°C), pH, electrical conductivity (*μ*S/cm), turbidity (NTU), TDS (mg/l), total hardness (mg/l), total alkalinity (mg/l), NO_3_-N (mg/l), PO_4_^3−^‐P (mg/l), NH_3_-N (mg/l), chlorides (mg/l), calcium (mg/l), magnesium (mg/l), sodium (mg/l), potassium (mg/l), iron (mg/l), DO (mg/l), COD (mg/l), BOD_5_ (mg/l), total coliform bacteria, chlorophyll-a (*μ*g/l), and salinity (%), were measured (Table 1).

Physicochemical and biological parameters will reveal the pollution status of the lake based on their concentrations. According to the previous studies, pH [16], temperature changes [17], dissolved oxygen [18], fertilizers [19], salinity [20], ammonia [21], algae [22], phosphates [23], drought conditions, and overcrowded fish populations are the major reasons for fish death in aquatic ecosystems. So the parameters mentioned in Table 1 were analyzed in the laboratory, and a minimum of 18 parameters are needed to calculate the water quality index [4].

### 2.5. Water Quality Indices

Water quality index (WQI) is one of the most effective tools to convey complex water quality information into a simple dimensionless value, which can be understood easily by authorities, decision-makers (policy-makers), and concerned communities [24]. Water quality indices incorporate data from multiple water quality parameters into a mathematical equation that provides a single number that expresses the overall water quality at a certain location and time. Each water quality index method has a rating scale to express the status of water quality concerning the index value of the lake at selected sampling points. This indexing method has seen widespread use since its commencement and was employed by multiple states and countries [25–27].

#### 2.5.1. Canadian Council Members of Environment (CCME) Water Quality Index

CCME WQI is one of the water quality indices to determine the status of water quality at various sampling points in the water body. The benchmark of a CCMEWQI is standards of water quality parameters or site-specific background concentration [28, 29]. The Canadian Council Member of the Environment (CCME) water quality index method has three factors, that is, scope (*F*1), frequency (*F*2), and amplitude (*F*3) to calculate the index of Chamo Lake at various sampling points. The number of tests failed tests and failed variables influence the water quality index results in CCMEWQI. The CCMEWQI scale was divided into five categories, namely, excellent, good, fair, marginal, and poor (Table 2).

(1) $$\begin{array}{c} \text{CCME WQI}=100–\left(\frac{\sqrt{F1^{2}-F2^{2}-F3^{2}}}{1.732}\right), \end{array}$$

where *F*1 = (no. of failed variables/total no. of variables) *∗* 100 and *F*2 =  no. of failed tests/total no. of tests) ^*∗*^ 100.

Find F3:

- excursion_i_ = (failed test value/objective_*j*_) − 1
- nse = no. of tests
- *F*3 = (nse/0.01nse + 0.01)

#### 2.5.2. US National Sanitation Foundation Water Quality Index (NSFWQI)

Brown et al. (1972) [30] developed a water quality index and elaborated Delphic exercises paying great rigour in selecting parameters, developing a common scale, and assigning weights. Rating curves were developed from questionnaire results of the experts on attribute values for variations in the level of water quality caused by different levels of the selected parameters [4, 31]. With the establishment of rating curves and associated weights, various methods of computing a water quality index are possible. The NSFWQI equation is mentioned as follows:

(2) $$\begin{array}{c} \text{NSFWQI}=\sum_{i=1}^{p}W_{i}Q_{i}, \end{array}$$

where *W*_*i*_ is the weightage associated with the *i*^th^ water quality parameter, *Q*_i_ is the subindex for i^th^ water quality parameters, and *P* is the number of water quality parameters.

The NSF water quality index category scale was mentioned in Table 2.

### 2.6. Statistical Analysis

Statistical analysis was done for water quality analytical results data to justify the accuracy and reliability of the primary data. SPSS was used for descriptive, correlation, and ANOVA tests. Descriptive statistics were used for mean computation. A correlation test has been carried out to assess the relations of physicochemical characteristics of lake water with its biological characteristics. In addition, one-way ANOVA was also used, and Origin 8.5 was employed for graphical illustrations.

## 3. Results and Discussion

### 3.1. Water Quality Results (Wet and Dry Seasons)

Twenty-two parameters were analyzed for the collected samples of Chamo Lake based on the standard methods [15]. The results are mentioned in Table 3 regarding five sampling points during both seasons. The concentrations of the parameters *pH*, temperature, BOD5, COD, total alkalinity, TDS, ammonia-nitrogen, and iron were higher than the permissible limits in both seasons. Total solids concentrations in the wet season and electrical conductivity and phosphates during the dry season were greater than the acceptable limits of WHO standards in Chamo Lake. The parameters that are above the permissible limit were discussed in detail.

#### 3.1.1. Temperature

The temperature in the Chamo Lake was in the range of 22.6–23.0 C during the wet season and 31.30–32.30 C during the dry season that are above the permissible limit of WHO standards (Table 3). Temperature plays a prominent role in dissolved oxygen levels because temperature establishes a maximum oxygen-holding capacity of water [32]. High water temperatures (86°F or higher) reduce the holding capacity. Untreated domestic wastewater causes to increase in the temperature of the water [33]. During the dry season, higher temperatures cause to increase in the evaporation rate leading to an augment in the concentration of pollutants in the water and decreasing the dissolved oxygen concentrations in the lake.

#### 3.1.2. Total Dissolved Solids (TDS)

Total dissolved solids concentration in Chamo Lake was in the range of 699–705.5 mg/L during the wet season, which is within the acceptable limit (Table 3). During the dry season, TDS results were recorded in the range of 1,082–1,093.7 mg/l, which is higher than the permissible limit of 900 mg/l. It might be the reason for higher temperatures to enhance the dissolving capacity of solids in the water [34].

#### 3.1.3. Total Alkalinity

Total alkalinity values in Chamo Lake were in the range of 630–678 mg/L during the wet season and 650–768 mg/L in the dry season, which is above the WHO permissible limit (Table 3). Higher concentrations of alkalinity might be the reason for the salts, which might be dissolved additional in higher temperatures in the dry season [32].

#### 3.1.4. Ammonia (NH4-N)

The concentration of ammonia in Chamo Lake samples is in the range of 14–19.6 mg/L during the wet season and 16.8–23.8 mg/L during the dry season, which was higher than the permissible limit of WHO standards (Table 3). The decomposition of organic matter releases ammonia in the form of unionized ammonia (NH_3_) or ionized ammonia (NH_4_^+^) [35, 36]. Unionized ammonia (NH_3_) is toxic to fish and lethal to increased water temperature and *pH* [37]. Ammonia concentrations of 7.40 mg/L were shown to cause mass mortality in tilapia fingerling within 24 h [38]. Higher concentrations of ammonia exposed by fish cannot excrete ammonia efficiently; as a result, ammonia levels in blood and tissues increase along with *pH* levels, thereby affecting enzyme activity [39]. These ammonia higher concentrations might be due to the untreated domestic wastewater and agricultural runoff water entering Chamo Lake. Sediment inflow also causes to increase in the NH_4_-N concentration in the lake [40].

The concentrations of ammonia in the lake were higher than the proposed threshold toxicity levels for tilapia with acceptable limits (less than 0.5 mg/L) at all sampling points [41]. The level of unionized ammonia, which has an impact on growth rate and can kill fish over a few days ranged between 0.2 and 0.6 mg/L [42], while the acute toxicity (24 h) of Nile tilapia fingerling is 7.4 mg/L [38].

#### 3.1.5. Phosphates

The concentration of phosphate in Chamo Lake was in the range of 0.30–0.39 mg/L during the wet season and 0.82–1.10 mg/L during the dry season, which is higher than the WHO permissible limit of <0.15 mg/l (Table 3). The highest concentration of phosphate was found at CH-05 where there is an agricultural inflow area of the lake. The higher concentrations of phosphates during the dry season might be the reason for evaporation, the inflow of agricultural runoff, and untreated domestic wastewater to the lake [2]. Phosphate concentration causes increased plant growth and reduces dissolved oxygen, which can lead to the death of fish as well [10].

#### 3.1.6. Iron (Fe)

The concentration of iron in the lake was in the range of 0.31–0.42 mg/L during the wet season and 0.53–0.64 mg/L during the dry season, which is higher than the WHO standard permissible limit of 0.30 mg/l (Table 3). The higher values of iron in the dry season might be the evaporation and reduction of inflow to dilute concentration. The highest concentration was found at CH-01 where the Kulfo River entered the lake. This highest value might be due to the untreated domestic wastewater and agricultural runoff water inflow to the lake [43].

#### 3.1.7. Dissolved Oxygen (DO)

The dissolved oxygen concentration in the lake was found in the range of 6.63–6.70 mg/L during the wet season and 5.20–5.52 mg/L during the dry season (Table 3), which is lesser than the permissible limit of >7 mg/l at 25°C as per the USEPA standards. These lower concentrations of dissolved oxygen might be the higher load of untreated wastewater, in addition to the higher concentrations of ammonia and higher temperatures in the lake. The Nile tilapia feed intake and growth will be reduced when the dissolved oxygen concentrations are lower than 3 mg/L [44]. These lower concentrations of dissolved oxygen in the lake may cause suffocation of aquatic life and the death of fish [2]. The reduced DO levels significantly increased the acute toxicity of ammonia to leader prawns (*Penaeus monodon*) [45].

Temperature and dissolved oxygen have interdependent parameters, as per the guidelines of USEPA. As per the range of temperature (22.6–32.3 C) in Chamo Lake, samples should have dissolved oxygen concentration of 8.8–8.5 mg/l minimum for the survival of aquatic life in the lake. All results of dissolved oxygen in Chamo Lake were in the range of 5.25–6.67 mg/L, which are below the acceptable limits. In many instances, fish mortality is directly owing to asphyxiation due to massively fallen dissolved oxygen levels [46]. In dry seasons, increased temperature results in a decrease in dissolved oxygen concentrations suddenly, which creates a shock to the aquatic life, and it may cause the death of fish in the lake.

#### 3.1.8. Biochemical Oxygen Demand (BOD)

The BOD values in the lake were in the range of 24.41–26.72 mg/L during the wet season and 35–38.52 mg/L during the dry season (Table 3), which is higher than the WHO standard permissible limit of 5 mg/l [15]. The highest BOD value was found at sampling point CH-01. This highest value might be due to the untreated domestic wastewater inflow to the lake. The greater the BOD, the more rapidly oxygen gets depleted in the water. The discharge of waste with higher levels of BOD can cause water quality problems such as severe dissolved oxygen depletion and fish kill in the receiving water bodies [47].

#### 3.1.9. Chemical Oxygen Demand (COD)

The chemical Oxygen Demand values in Chamo Lake were in the range of 64–76 mg/L during the wet season and 92–106 mg/L during the dry season, which is above the permissible limit of 10 mg/L as per the WHO standards (Table 3). The highest COD values were recorded where the untreated domestic wastewater entered the lake. The higher concentrations of COD in the lake might be due to urban wastewater and agricultural runoff, which will affect the aquatic life defectively [1]. The excessive amount of organic substances and metal ions in freshwaters generally originate from domestic sewage, urban runoff, industrial effluents, and farm wastes, which are the main causes of water pollution [48].

#### 3.1.10. Chlorophyll-a

Chlorophyll-a concentrations at sampling points CH-01, CH-02, CH-03, CH-04, and CH-05 in Chamo Lake were 31.87, 25.17, 24.65, 26.65, and 19.64 *μ*g/L during the dry season and 33.28, 27.43, 26.73, 28.38, and 31.87 *μ*g/L during the wet season, respectively (Table 3). All samples were having a high concentration of chlorophyll-a during the dry season [49], which is higher than the acceptable limit. The results depicted sampling points CH-01 (dry and wet seasons) and CH-05 (wet season) in the lower hypereutrophic state, sampling points CH-02, CH-03, and CH-04 (dry and wet seasons) in the eutrophic state, and sampling point CH-05 (dry season) in the fully eutrophic state.

The high levels of nutrients from fertilizers (agricultural runoff), organic matter (domestic wastewater), and turbidity (soil erosion) might be the reason for the high concentrations of chlorophyll-a, which indicates the presence of algal blooms [49, 50]. High biomass of plankton or suspended particles in the surface layer limits light penetration to the lower water layers [51].

#### 3.1.11. Salinity

The salinity of Chamo Lake was in the range of 0.70–0.93%, which is indicating the lake's salinity condition. Salinity in Chamo Lake was higher percentages; it might be due to the sediment inflow and increased concentrations of salts, and evaporation rate might be the reason for the higher concentrations in the dry season [52] in Chamo Lake.

Electrical conductivity and phosphates were above the acceptable limits in the dry season, but in the wet season, these were within the WHO standard permissible limits, which might be the reason for dilution by floodwater. As per the results, total solids were very high in concentration in the wet season than in the dry season. It might be the reason for high sediment inflow through Kulfo, Sele, and Elgo Rivers during the wet season in the lake (Table 4). Chamo Lake samples have high concentrations of organic matter (BOD and COD) and nutrients (phosphates and nitrates); these might be untreated domestic wastewater through Kulfo, Sele, and Elgo Rivers into the lake (Figure 3) [53]. The high content of organic matter, nutrients, and chlorophyll-a concentrations leading to the low dissolved oxygen content in the lake might be caused for the suffocation of the fish as well as eutrophication [54].

The accuracy of the water quality results was analyzed with the help of statistical analysis and one-way ANOVA to know the rejection or acceptance of the null hypothesis. If the null hypothesis is true, *F* values will be closed to 1.0 most of the time. High *F*-values indicate the null hypothesis rejection. The high *F*-value graph shows a case where the variability of group means is large relative to the within-group variability (Figure 4). This means the influence of parameters on water quality is very highly acceptable.

### 3.2. Chamo Water Quality Index

The Canadian Council Member of Environment (CCME) water quality index results at all sampling points (CH-01, CH-02, CH-03, CH-04, and CH-05) in both the dry and wet seasons were in the range of 13.90–18.40, which are in the category of “poor.” The most influential 18 parameters out of 20 parameters were taken for the calculation of the Canadian Council Members of Environment (Table 4).

All Canadian Council Members of Environment (CCME) results were “poor” that was influenced by the number of failed parameters and failed tests. Firstly, the failed parameters were in the range of 15–16 out of 18 parameters; this might be the reason for the result of the water quality index category “poor.” During the dry season, water quality index results were found higher than the wet season index results. It might be due to high temperatures as well as the absence of flood inflow to dilute the concentration of pollutants [55]. Sampling point CH-01 has the highest index results were identified. The sampling point CH-01 is located where the Kulfo River drains into Chamo Lake. In the dry season, water quality index results were influenced by high concentrations of pH, electrical conductivity, temperature, turbidity, BOD5, COD, phosphates, ammonia-nitrogen, and total coliform bacteria (APHA 2005). This index was designated as the water quality of Chamo Lake at all sampling points was “poor” (Table 4). This indicates the Chamo Lake water will not be useful for drinking as well as harmful to aquatic life.

Secondly, the failed tests were in the range of 54–60 (83.33–88.88%) out of 72, influencing CCME water quality index results of Chamo Lake water samples. The failed test means the parameter's results are above the acceptable limits of the WHO standards. These might be influenced by failing parameters and failed tests of Chamo Lake water samples. The nse values were in the range of 5.55–6.23.

NSFWQI method was also used to confirm the water quality of Chamo Lake, in addition to CCMEWQI. The results were mentioned in Table 4. The NSF water quality index results at all sampling points were in the water quality category of “bad” (38.59–49.63) in both seasons (Table 5). During the wet season, the water quality category values are very close to the “medium” category.

As per the results, we found that in the wet season, index values were close to medium rather than in the dry season index results. NSFWQI results were in the range of 38.59–45.11 during the dry season and 48.12–49.63 during the wet season, which is very close to the medium range of 51–70. This might be due to the dilution effect of floodwater in the wet season. NSFWQI category “bad” indicates lake water is unfit for drinking purposes and harmful to aquatic life. Two indices (CCMEWQI and NSFWQI) confirmed that the water quality of Chamo Lake is not suitable for drinking.

### 3.3. Water Quality Control Measures for Chamo Lake

Three rivers (Kulfo, Sele, and Elgo) and agricultural runoff draining into Chamo Lake were observed. Tourists are visiting the lake regularly. These were identified as possible pollution sources of Chamo Lake by satellite data images delineated using ArcGIS (Figure 3). The inflow of the Kulfo River that was higher than the inflow of Sele and Elgo rivers into the lake was observed in both seasons. The control of pollutants from the Kulfo, Sele, and Elgo Rivers can protect the quality of Chamo Lake. In the peripheral region of the lake, excess plant growth was observed. Preparation of guidelines for tourists to dispose of waste properly and safely as well as strict enforcement of the guidelines will control the pollution from tourists.

#### 3.3.1. Agricultural Runoff Water

Treatment facility establishment of agricultural runoff water will be difficult. So other alternative methods such as construction of the bund or teras near the lake and drip irrigation should be implemented to reduce or minimize the agricultural runoff water into the lake as well as to control the wastage of water [56].

#### 3.3.2. Sediment Control

Sediment is the major problem to increase the turbidity of water and causes to siltation effect in the draining lakes, finally vanishing from lakes. This sediment can control by growing the grass or plants along the lake peripheral region to reduce or minimize the sediment inflow and soil erosion. Bend-way weirs can construct to control the flow at bending areas: Stone weirs are one of the best methods to control the sediment into the lake at inlet areas. These stone weirs can arrange across the Kulfo, Sele, and Elgo rivers before the inlet of Chamo Lake can control the sediment inflow.

## 4. Conclusion

Chamo Lake has higher concentrations of organic matter (COD and BOD), nutrients (phosphates and iron), chlorophyll-a, pH, EC, TDS, turbidity, alkalinity, salinity, ammonia, and *Escherichia coli* bacteria were identified through water quality analysis. Dry season concentrations of pollutants were higher than the wet season concentration except for turbidity and *E. coli* bacteria due to high temperatures might be caused higher evaporation. The highest concentrations of turbidity and *E. coli* in the wet season were found due to sediment inflow by floodwaters (soil erosion) and urban floodwaters. The death of fish in the lake during the dry season was due to higher concentrations of ammonia, temperature, and sudden reduction of dissolved oxygen. According to the CCME and NSF, water quality indices concluded the general quality status of Chamo Lake was “poor” in both seasons and “bad” in the dry season plus all sampling points were close to “medium” in the wet season. The status of Chamo Lake is harmful to domestic purposes and aquatic life but useful for irrigation purposes. The sources of pollutants were found that untreated domestic wastewater through Kulfo, Sele, and Elgo rivers, agricultural runoff, sediment inflow, and urban floodwater by the survey. Future research can concentrate on sediment load assessment, sediment chemical composition, and design of structures for controlling sediment inflow that will give more appropriate solutions for lake sustainability.

## Figures and Tables

**Figure 1:** Location map of the study area of Chamo Lake.

**Figure 2:** Annual averages of rainfall and temperature at the study area.

**Figure 3:** Major pollution sources of Chamo Lake.

**Figure 4:** Water quality parameters with *F*-values during both dry and wet seasons.

**Table 1:** Analytical methods and instruments used for various water quality parameters.

Parameter	Analytical method	Instrument used (name and model)
Temp (°C), pH, electrical conductivity (*μ*S/cm), salinity, DO (mg/l)	Digital multiparameter analyzer	Multimeter (HQ40 d, USA)
Turbidity (NTU)	Nephalometric	Turbidity meter, HACH 2100A
TDS (mg/l)	Gravimetric	Oven dry, Memmert 854 Schwabach
Total hardness as CaCO_3_ (mg/l), calcium (mg/l), and magnesium (mg/l)	EDTA titrimetric	Titration setup
Total alkalinity as CaCO_3_(mg/l)	Titrimetric	Titration setup
NO_3_-N (mg/l), PO_4_^3−^‐P (mg/l), chlorophyll-a (*μ*g/l)	Spectrophotometric	UV-VIS spectrophotometer, Systonic, India
NH_3_-N	Colorimetric	Distillation setup
Chloride (mg/l)	Argentometric	Titration setup
Fluorides	SPADNS	DR-2800 (HACH, USA)
Potassium (mg/l)	Flame photometry	Dual channel flame photometer, model-2655-10
Iron (mg/l)	Spectrophotometric	DR-2800 (HACH, USA)
Chemical oxygen demand (mg/l)	Open reflex	CSB thermostat
Biological oxygen demand (BOD_5_) (mg/l)	Modified Winkler	BOD incubator set at 20°C, Memmert, west Germany 854 Schwabach
Total coliform bacteria	Membrane filtration	Incubator set at 37°C, Memmert, west Germany

**Table 2:** Water quality indexes and scales.

Canadian Council of Ministers of the Environment water quality index		US National Sanitation Foundation water quality index	
Water quality index value	Rating of the water quality	Water quality index value	Rating of the water quality

95–100	Excellent	90–100	Excellent
80–94	Good	71–90	Good
60–79	Fair	51–70	Medium
45–59	Marginal	26–50	Bad
<44	Poor	0–26	Very bad

**Table 3:** Chamo Lake water samples analytical data in both the dry and wet seasons.

Parameter	Chamo Lake water quality analytical results at five sampling points									
CH-01		CH-02		CH-03		CH-04		CH-05	
Dry	Wet	Dry	Wet	Dry	Wet	Dry	Wet	Dry	Wet
Temp (°C)	32.30 ± 0.49	22.7 ± 0.59	32.20 ± 0.49	23.0 ± 0.59	32.30 ± 0.49	22.70 ± 0.59	32.30 ± 0.49	23.0 ± 0.59	31.3 ± 0.49	22.6 ± 0.59
pH	9.10 ± 0.19	8.90 ± 0.26	9.20 ± 0.19	9.00 ± 0.26	9.20 ± 0.19	9.00 ± 0.26	9.20 ± 0.19	9.00 ± 0.26	9.30 ± 0.19	9.00 ± 0.26
EC (*μ*S/cm)	1,702 ± 10.86	1,409 ± 2.75	1,705 ± 10.86	1,408 ± 2.75	1,692 ± 10.86	1,411 ± 2.75	1,715 ± 10.86	1,407 ± 2.75	1,708 ± 10.86	1,404 ± 2.75
TDS (mg/l)	1,087 ± 5.45	702 ± 2.9	1,089.5 ± 5.45	704 ± 2.9	1,082 ± 5.45	705.5 ± 2.9	1,093.5 ± 5.45	703.5 ± 2.9	1,090 ± 5.45	699 ± 2.9
Total hardness (mg/l)	60 ± 2.6	60 ± 8.03	56 ± 2.6	50 ± 8.03	54 ± 2.6	70 ± 8.03	56 ± 2.6	50 ± 8.03	54 ± 2.6	74 ± 8.03
Total alkalinity as CaCO_3_ (mg/l)	730 ± 34.8	630 ± 18.6	650 ± 34.8	640 ± 18.6	750 ± 34.8	660 ± 18.6	716 ± 34.8	660 ± 18.6	768 ± 34.8	678 ± 18.6
NO3-N (mg/l)	1.30 ± 0.26	1.24 ± 0.13	0.67 ± 0.26	0.94 ± 0.13	0.92 ± 0.26	0.90 ± 0.13	0.76 ± 0.26	0.90 ± 0.13	0.74 ± 0.26	0.95 ± 0.13
PO_4_^3−^‐P (mg/l)	0.82 ± 0.10	0.39 ± 0.04	0.89 ± 0.10	0.31 ± 0.04	0.98 ± 0.10	0.30 ± 0.04	0.91 ± 0.10	0.31 ± 0.04	1.10 ± 0.10	0.34 ± 0.04
NH3-N	23.80 ± 2.8	14.00 ± 3.29	19.60 ± 2.8	16.80 ± 3.29	23.80 ± 2.8	15.40 ± 3.29	16.80 ± 2.8	14.25 ± 3.29	21.00 ± 2.8	19.60 ± 3.29
Chloride (mg/l)	234.00 ± 3.75	200.7 ± 3.41	238.0 ± 3.75	192.7 ± 3.41	231.00 ± 3.75	196.70 ± 3.41	231.00 ± 3.75	196.70 ± 3.41	238.00 ± 3.75	191.67 ± 3.41
Sulfates (mg/l)	45.00 ± 2.09	58.72 ± 8.95	42.00 ± 2.09	39.15 ± 8.95	41.00 ± 2.09	38.30 ± 8.95	43.00 ± 2.09	58.72 ± 8.95	45.00 ± 2.09	37.45 ± 8.95
Calcium (mg/l)	14.00 ± 1.04	20.40	14.40 ± 1.04	22.03	14.00 ± 1.04	22.85	14.00 ± 1.04	22.08	16.00 ± 1.04	21.22
Magnesium (mg/l)	11.30 ± 0.85	9.62 ± 2.22	10.10 ± 0.85	6.80 ± 2.22	10.00 ± 0.85	11.46 ± 2.22	10.30 ± 0.85	11.46 ± 2.22	9.20 ± 0.85	12.83 ± 2.22
Iron (mg/l)	0.64 ± 0.05	0.42 ± 0.04	0.55 ± 0.05	0.32 ± 0.04	0.57 ± 0.05	0.35 ± 0.04	0.53 ± 0.05	0.42 ± 0.04	0.54 ± 0.05	0.31 ± 0.04
DO (mg/l)	5.28 ± 0.26	6.70 ± 0.20	5.20 ± 0.26	6.67 ± 0.20	5.52 ± 0.26	6.65 ± 0.20	5.25 ± 0.26	6.67 ± 0.20	5.32 ± 0.26	6.63 ± 0.20
COD (mg/l)	104.00 ± 6.2	66.00 ± 3.97	92.00 ± 6.2	64.00 ± 3.97	106.00 ± 6.2	76.00 ± 3.97	102.00 ± 6.2	64.00 ± 3.97	92.00 ± 6.2	70.00 ± 3.97
BOD_5_ (mg/l)	38.52 ± 2.29	25.38 ± 1.44	36.28 ± 2.29	24.61 ± 1.44	37.14 ± 2.29	25.23 ± 1.44	35.00 ± 2.29	24.41 ± 1.44	36.00 ± 2.29	26.72 ± 1.44
Chlorophyll-a (*μ*g/l)	31.87 ± 3.88	33.28 ± 2.88	25.17 ± 3.88	27.43 ± 2.88	24.65 ± 3.88	26.73 ± 2.88	26.65 ± 3.88	28.38 ± 2.88	19.64 ± 3.88	31.87 ± 2.88
Salinity (%)	0.92 ± 0.01	0.70 ± 0.01	0.93 ± 0.01	0.7 ± 0.01	0.91 ± 0.01	0.70 ± 0.01	0.93 ± 0.01	0.7 ± 0.01	0.93 ± 0.01	0.70 ± 0.01

**Table 4:** Canadian Council Members of Environment water quality index results of Chamo Lake.

Sampling station	Season	*F*1	*F*2	*F*3	nse	Number of total tests	Number of failed tests	Number of passed tests	CCMEWQI	WQI category
CH-01	Dry	88.88	83.33	85.95	6.12	72	60	12	13.90	Poor
	Wet	83.33	79.16	85.17	5.74	72	57	15	17.40	Poor

CH-02	Dry	83.33	76.38	84.80	5.58	72	55	17	18.40	Poor
	Wet	88.88	75.00	85.69	5.99	72	54	18	16.59	Poor

CH-03	Dry	88.88	77.77	85.46	5.88	72	56	16	15.82	Poor
	Wet	83.33	77.77	84.73	5.55	72	56	16	17.99	Poor

CH-04	Dry	83.33	77.77	85.69	5.99	72	56	16	17.66	Poor
	Wet	83.33	77.77	85.00	5.67	72	56	16	17.89	Poor

CH-05	Dry	88.88	79.16	85.99	6.14	72	57	15	15.22	Poor
	Wet	83.33	77.77	86.17	6.23	72	56	16	17.49	Poor

**Table 5:** National Sanitation Foundation water quality index of the Chamo Lake.

Sample	Season	Temp	*pH*	Turbidity	Nitrate	Phosphates	Total solids	DO	BOD5	Total coliform	Total WQI
Wi	0.10	0.11	0.08	0.1	0.1	0.07	0.17	0.11	0.16
CH-01	Dry	Qi	18.5	47	49.2	93.5	50.8	20	31.256	2	39.2	
		WQI	1.85	5.17	3.936	9.35	5.08	1.4	5.3135	0.22	6.272	38.59
	Wet	Qi	18.84	51	21	93.8	76.6	20	85.60	7	32.4	
		WQI	1.884	5.61	1.68	9.38	7.66	1.4	14.55	0.77	5.184	48.12

CH-02	Dry	Qi	18.3	42.4	58.4	96.65	46.6	20	55	2	40.84	
		WQI	1.83	4.664	4.672	9.665	4.66	1.4	9.35	0.22	6.534	42.99
	Wet	Qi	18.8	48	23.4	95.3	81.4	20	85	5	39.28	
		WQI	1.88	5.28	1.872	9.53	8.14	1.4	14.45	0.55	6.285	49.38

CH-03	Dry	Qi	17.52	42.4	61.8	95.4	41.2	20	68.86	2	42.28	
		WQI	1.752	4.664	4.94	9.54	4.12	1.4	11.71	0.22	6.76	45.11
	Wet	Qi	19.4	48	36.6	95.5	82	20	85.2	2	35.2	
		WQI	1.94	5.28	2.93	9.55	8.2	1.4	14.48	0.22	5.63	49.63

CH-04	Dry	Qi	17.52	42.4	59.2	96.2	45.4	20	64	2	40.12	
		WQI	1.752	4.66	4.74	9.62	4.54	1.4	10.88	0.22	6.42	44.23
	Wet	Qi	18.8	48	31.8	95.5	81.4	20	85	5	34	
		WQI	1.88	5.28	2.54	9.55	8.14	1.4	14.45	0.55	5.44	49.23

CH-05	Dry	Qi	17.52	39.6	60	96.3	38.8	20	65.5	2	40.88	
		WQI	1.752	4.356	4.8	9.63	3.88	1.4	11.14	0.22	6.54	43.71
	Wet	Qi	29.8	48	29.8	95.25	79.6	20	84.34	2	33.87	
		WQI	2.384	5.28	2.384	9.525	7.96	1.4	14.34	0.22	5.42	48.42

## Data Availability

Data will be made available at a reasonable request.
